This article has been retracted.

# Assessment of Bacterial Isolates from the Urine Specimens of Urinary Tract Infected Patient

**DOI:** 10.1155/2022/4088187

**Published:** 2022-07-27

**Authors:** Chennu M. M. Prasada Rao, T. Vennila, Sreya Kosanam, P. Ponsudha, K. Suriyakrishnaan, Abdullah A. Alarfaj, Abdurahman Hajinur Hirad, S. R. Sundaram, P. A. Surendhar, Nagarajan Selvam

**Affiliations:** ^1^Department of Pharmaceutical Chemistry, School of Pharmacy, Raffles University, Neemrana, Rajasthan 301020, India; ^2^Department of Chemistry, Sri Sairam Engineering College, Chennai, Tamil Nadu 602109, India; ^3^Department of Pharmacology and Pharmacy Practice, Nirmala College of Pharmacy, Atmakur, Andhra Pradesh 522503, India; ^4^Department of Electronics and Communication Engineering, Velammal Engineering College, Chennai, Tamil Nadu 600066, India; ^5^Department of Electronics and Communication Engineering, Sona College of Technology, Salem, Tamil Nadu 636005, India; ^6^Department of Botany and Microbiology, College of Science, King Saud University, P.O. Box 2455, Riyadh 11451, Saudi Arabia; ^7^Department of Sciences, University of Tennessee Health Science Center, Memphis, TN 38103, USA; ^8^Department of Biomedical Engineering, Vels Institute of Science, Technology and Advanced Studies (VISTAS), Chennai, Tamil Nadu, India; ^9^Department of Computer Science, Ambo University, Ethiopia

## Abstract

Urinary tract infections (UTIs) maintained a serious public health concern, as did the growth in antibiotic resistance both between uropathogenic microorganisms. A regular assessment of the microbiological agents that cause UTIs, as well as their antimicrobial resistance, is essential for a tailored empirical antibiotic response. Knowing the variables that cause UTIs can help you intervene quickly and simply to get the condition under control. The most common infecting species in acute infection is Escherichia coli (E. coli). To strengthen infection control strategies, it is necessary to know the prevalence and location of UTI. The goal of this research is to measure the frequency of microorganisms isolated from patients with UTIs as well as the antimicrobial sensitivity characteristics of Gram-negative bacteria. The purpose of this research has been to evaluate the frequency of UTIs by extracting and characterizing the various bacterial etiological organisms, as well as to assess the factors linked to UTIs. The goal of this research is to identify, characterize, and establish the antibiotic susceptibility patterns of bacteria linked to urinary tract infections. Fresh collected urine specimen was taken from inpatients or outpatients in UTI cases and bacteriologically tested using conventional microbiological methods. The Kirby-Bauer disc diffusion method was used to create the antibiogram. Staphylococcus saprophyticus, Staphylococcus aureus (28%), and Escherichia coli (24.6%) were the most common isolates (20%). The evaluated agents' antibacterial activity was all in the following order: cefixime, ciprofloxacin, augmentin, gentamicin, ceftazidime, nitrofurantoin, ofloxacin, and cefuroxime. It was discovered that each and every one of the microbes exhibited varied degrees of resistance to the antibiotics nitrofurantoin, ciprofloxacin, and ofloxacin. Every type of bacteria, with the exception of those belonging to the genus Streptococcus, has a Multiple Antibiotic Resistance Index (MARI) that is more than 0.2. The first-line therapies for urinary tract infections (UTIs) in the region would consist of ciprofloxacin, ofloxacin, and nitrofurantoin. Lower urinary tract infections almost never result in problems if they are diagnosed and treated as soon as possible and in the correct manner. However, if treatment is not sought, a urinary tract infection can lead to serious complications.

## 1. Introduction

The microbial infection of any region of a urinary tract is referred to as a urinary tract infection (UTI). It is between the most frequent bacteriological infections in both men and women, with a feminine predisposition. Antibiotics are frequently used to detect and cure infectious diseases; however, some bacteria have evolved the ability to thrive in an antibacterial drug environment, resulting in “antibiotic resistance.” Sexual activity, vaginal infections, antimicrobial activities of prostatic fluids, diabetes, hygiene practices, obesity, and genetic predisposition are all risk factors for UTIs [1]. The diagnosis is made by combining a urine culture with both the existence of clinical symptoms, and antimicrobial sensitivity is assessed by diffusion method, dilution testing, and the death curve. Serratia, Gram-negative rods, Proteus spp., Klebsiella, Enterobacteriaceae, Pseudomonas aeruginosa, Gram-positive cocci included enterococci, and other organisms such as Candida spp. are the most frequent uropathogens, accounting for 80% of the community-acquired illnesses and 40% of the nonsocietal infections. It is crucial to be aware of this to achieve high cure rates and low resistant levels [2]. Nevertheless, antimicrobial resistance is improving at an alarming rate around the world. Antimicrobial resistance is caused by overuse, inappropriate prescribing, and scarcity of novel antibiotics and regulatory hurdles. As a result, enforcing antibiotic-monitored regimens is beneficial in reducing the risk of resistant bacteria.

There is average of entering a postantibiotic era, during which common infections will no longer be treated with antibiotics. In 2013, the Centers for Diseases Management and Prevention recommend that every year around millions of people were infected through antibiotic-resistant bacterium [3]. Antibiotic susceptibility is increasing in all age groups; hence, investigating common infections and assessing their antibiotic susceptibility are critical. Resistance to antibiotics is a worldwide and local concern in Iraq, endangering dozens of lives, particularly in low-income or conflict-affected communities. “The future of humanity and germs will certainly evolve as the events of wits vs. their genes,” predicted Nobel laureate Joshua Lederberg roughly 19 years ago. Excluding the distal urethral, which is colonized by saprophyte microorganisms from the surrounding countryside, the urinary system is a sterile space; hence, a urine sample acquired by peeing is not regarded as a basic healthy sample [4]. Once an infection has taken hold in the bladder, germs can quickly multiply and reach high quantities in the urine, allowing them to thrive. Microorganisms could enter the urinary system through blood flow or lymphatic enlargement, and there is evidence of experimental and clinical data to suggest that bacteria from the urethra are perhaps the most mutual source of UTI, particularly bacteria from an intestine.

The greatest category of specimens studied in healthcare microbiology laboratories is urine collection microscopy, cultures, and sensitivities that offer verification in the medicinal utilization of antibiotics. Furthermore, across all areas of healthcare administration, the clinical perception of UTI seems to be the second most popular criterion for empirical antibiotic therapy [1]. The growth in uropathogenic microorganisms resistant to presently used antibiotics is a distinct major concern as in empirical utilization of antibiotics among patients with UTI around the world. This is although there have been fewer breakthroughs in the discovery of novel antibiotics. It was discovered that even a sure enough empirical therapy of illnesses is one strategy to suppress resistance to antibiotics [5]. In most parts of the poor world, detailed data on uropathogenic microorganisms and their trends of susceptibility and resistance are typically unavailable or outdated, as antibacterial susceptibility profiles are bound to vary over time. As a result, a periodic review of the microbial pathogens of UTIs, as well as their antibacterial resistance, is indeed desirable, but also necessary for a tailored empirical antibiotic treatment in patients with suspected UTIs.

The majority of uropathogens of healthy people come from the rectal bacteria and reach the urinary tract through the urethra into the bladder. Uropathogens first attach to and populate related to the local of a proximal urethra via the ascending route as in Figure 1. Individuals with staining from around the lower abdomen, patients having urinary catheters, or females who take spermicidal drugs have a harder time enhancing this channel [6]. Up to 50% of illnesses in individuals with established cystitis could ascent through into higher urinary tracts, and also, the majority of instances of pyelonephritis were associated with increased morbidity ascending from the bladder over all the ureter and then into the renal pelvis [7]. Bacterial ascent is helped by situations that impede ureteral peristalsis, including pregnancies and ureteral blockage. Bacteria which enter the renal pelvis into the gathering ducts can infiltrate the renal tissues and damage the renal tubules.

It is among the greatest prevalent bacterial infections encountered in a clinical practice, especially in developing nations, with a high percentage of morbidity and economic cost. Poor hygiene practices and urinary system abnormalities have been identified as some of the primary variables that predispose to UTI. The agents that cause UTI differ from one location to the next, as do their sensitivity and development of resistance [8]. Various bacterial pathogens are responsible for UTIs. Staphylococcus saprophyticus, Escherichia coli, Staphylococcus aureus, Klebsiella pneumoniae, Proteus sp., enterococci, and Pseudomonas aeruginosa seem to be the most prevalent pathogenic organisms associated with UTI [9]. Treatment for urinary tract infections is frequently initiated on an empirical basis, with information derived from the antibiotic resistance characteristic of the urine pathogens. Despite the development and use of antimicrobial medications, the number of UTIs produced by infection has been rising in recent years. The rise has been attributed in part to the emergence of antibiotic sensitivity across urinary tract infections. Resistant bacteria in microbial uropathogens are a significant and rapidly increasing public health issue. Antibiotic resistance to urinary pathogens is on the rise all around the world.

UTIs become more common as people become older, with 25-50% of females aged 80 and up having bacteriuria. UTIs are caused by interactions among the uropathogen as well as the host, and their aetiology is complicated. The uropathogenic pathogen first adheres to the epithelial surface before colonizing and disseminating all across the mucosa, producing tissue destruction [10]. Pathogens can climb into the urine bladder after the original colonization era, causing symptomatic or asymptomatic bacteriuria. Pyelonephritis and renal disease may develop if the condition worsens. Microbial resistance towards the host's ordinarily effective protective factors is caused by detailed virulency issues found on a uropathogen cell. Bacterial autoantibodies and related epithelium binding ability were recently discovered, and natural antiadherence systems are actively being researched.

When sensitivity characteristics are revealed, accurate microbiological records of cultural context offer recommendations on empirical therapy [11]. Because most UTIs are managed on a case-by-case basis, antimicrobial drug selection criteria should be created on the maximum likely infection and its projected resistance trend in a given geographic area. As a result, there is no requirement to monitor the contributing organism of UTI and associated resistance patterns in a given area regularly. In Awka, the resistance patterns of community-acquired uropathogens have not remained thoroughly investigated. There has been no documentation of resistant bacteria in UTIs with Amaku yet. As a result, the goal of this study is to identify bacterial uropathogens including their antibiotic sensitivity characteristics across UTI patients in Awka.

## 2. Related Work

This study comprised 440 culture-positive isolated bacteria among 1110 urine samples provided over a year. The usual biochemical analysis of the species was used to identify the isolated bacteria. The disc diffusion method was used to test the antibiotic susceptibility of culture-positive bacterial samples, as specified. 152 (34.6%) of the 440 culture-positive urine tests have been from interior people, while 288 (65.4%) came from outside sick people. Gram-negative bacteria made up 415 (95%) of the total isolates, whereas Gram-positive bacteria made up the remaining 27 (6%). P. aeruginosa 54 (12%) and Escherichia (E.) coli 270 (61.4%) have been the most common bacterial isolate, trailed by Pseudomonas and Klebsiella (K.) pneumoniae 42 (9.5%). E. coli (96.2%) isolates were susceptible to imipenem, 85.2% to amikacin, 80.7% to piperacillin/tazobactam, and 72.6% to nitrofurantoin, according to the susceptibility pattern. P. aeruginosa isolates were responsive to tazobactam/piperacillin in 73% of cases, sulbactam/cefoperazone in 69.2% of cases, and imipenem in 65.38% of cases. According to the antibiogram of K. pneumoniae, 76.2% of the bacteria were susceptible to imipenem and 52.3% to piperacillin/tazobactam. Antibiotics such as nitrofurantoin and imipenem were the maximum efficient against Enterococcus spp., with 92.3% showing sensitivity towards these isolated bacteria. The proportion of isolated bacteria was susceptible to imipenem and piperacillin/tazobactam, but susceptibility to the majority of routinely used oral medications was modest. Nitrofurantoin, between the oral antimicrobics, exhibited better sensitivity to Enterobacteriaceae and the Gram-positive microorganisms. However, the bulk of the samples was susceptible to imipenem and piperacillin/tazobactam, restricting the usage of popular UTI antibiotics [12].

However, it is unknown genetic variation in such animal representations relates to UPEC expression of genes in humans following UTI. To address this, employ a UPEC strain CFT073-specific microarray to evaluate global gene appearance in E. coli separates isolated immediately from urine of eight women who had bacteriuria and presented to a clinic. Ex vivo gene expression levels with the same E. coli isolates grown dynamically to exponential growth stage in collective, sterilized human urine were examined to those of the same E. coli infections cultured dynamically to exponential growth phase in aggregated, sterilized human urine. Known success factors such as iron uptake and peptide transport systems were strongly stated in human UTI, indicating that UPEC multiplies quickly in vivo. While all these results were typically similar to previous studies from the murine UTI models, there were some host-specific variations. However, it is unknown how genetic variation in such animal models relates to UPEC expression of genes in humans following UTI. To address this, employ a UPEC strain CFT073-specific microarray to evaluate global gene expression in eight E. coli isolates isolated immediately from the urine of women who had bacteriuria and presented to a clinic. Ex vivo gene expression levels with the same E. coli isolates grown dynamically to exponential growth stage in shared, purified human urine were examined the same E. coli infections educated dynamically to exponential growth phase in aggregated, sterilized human urine. Known success issues such as iron uptake and peptide transportation schemes are strongly uttered in human UTI, indicating that UPEC multiplies quickly in vivo. While all these results were typically similar to previous studies from the murine UTI models, there were some host-specific variations [13].

To find the common bacteria from probable urinary tract infections and how resistant they are to antibiotics, from 2003 to 2010, the Dessie Regional Laboratory performed a retrospective examination of pathogenic bacteria and their antibiotic susceptibility using urine tests. Antimicrobial sensitivity analyses were completed utilizing the disc diffusion approach, following the Kirby-Bauer method as a guideline. The patients are separated into two categories: males and females, with a male-to-female ratio of 1 : 1.96.319 (22.7%) of the total 404 samples tested positive for bacteria. The most common isolate was E. coli (63.7%), followed by Proteus spp. (8.2%) and Klebsiella spp. (8.5%). Overall, 85.6%, 88.9%, and 76.7% of bacteria were resistant to erythromycin, amoxicillin, and tetracycline, correspondingly. The three most common bacterial isolates displayed resistance to amoxicillin and tetracycline of 80.1% to 90.0% and susceptibility to ciprofloxacin, gentamicin, and nitrofurantoin of 25%. Antibiogram analysis revealed that 152 isolates (47.85%) were resistant to two or more antimicrobial drugs. Resistance to tetracycline, erythromycin, and amoxicillin was significant in the research area. Because the majority of isolates were responsive to gentamicin and nitrofurantoin, these antimicrobials were recommended for empirical treatment of urinary tract infections. In future research, a detailed age range is chosen for a group of urine tests [14].

Urinary tract infections (UTIs) in kids seem to be easy and basic, but there is still no agreement on UTIs under this patient population because it is one of the most—and not the most—contentious areas of pediatric healthcare. Many topics, particularly the diagnostic and therapy of UTIs in patient populations, are fraught with debate and absence of agreement. As a result, children with UTI are evaluated and managed in a variety of ways in different regions of the world, including within the same nation. The unanticipated difficulty in identifying UTI in youngsters is one element leading to the current predicament. This problem has ramifications not only for therapeutic practice but for scientific research. Practical challenges in at least three aspects, involving obtaining urine samples, properly assessing bacterial counts, and confounding infantile symptoms with a real acute febrile UTI, can lead to significant over- and underdiagnosis. These issues will be examined in-depth in this study and also the ramifications they may have on clinical settings and UTI study. Discuss a variety of significant topics related to UTI detection, with a special emphasis on bacteremia, which should be provided more consideration in future research [15].

The maximum prevalent source of E. coli bloodstream infections (BSI) is urinary tract infections; however, the process of bloodstream invasion remains unknown. At physiological temperatures, several clinical isolates were seen to protect themselves using extracellular amyloid filaments called curli. Curli fiber assembly at 37°C enhances bacteremia development in urinary E. coli strains, according to hypothesis. Curli expression in cultured E. coli isolated from bacteriuric individuals was studied utilizing Western blotting after amyloid fiber destruction with hexafluoroisopropanol within the condition and condition of bacteremia. Urinary samples isolated from bacteremia patients were much more effective than average individuals to express curli at 37°C [16/22 (73%) vs. 7/21 (33%); *p* = 0.01]. At 30°C, there was no substantial difference for curli expression 30°C [86% (19/22) vs. 76% (16/21)]. Patients' samples are clonally heterogeneous, showing that this trait is found in multiple generations. The majority of urine and blood isolated from the same patients are highly linked, indicating that urinary bacteria had entered the bloodstream directly. In this cohort, 37°C curli production was linked to bacteremia development of urinary E. coli isolates. The results point to new diagnostics and virulence-targeting treatment strategies in the future [16].

## 3. Materials and Methods

### 3.1. Study Design

Inpatient and outpatient care at Anambra State University Teaching Hospital in Amaku, Awka, is given clean-catch urine specimens. This sampling location was chosen since it encompasses the city's urban region. The study lasted four months (from April to August 2015). The research was conducted at Nnamdi Azikiwe Institution's Agulu Campus, Awka, at the Microbiology Lab of the Branch of Pharmaceuticals Microbiology and Biotechnology, Institute of Pharmaceutical Sciences.

To remove contaminants, the clean-catch technique was implemented to collect samples. Every patient's fresh collected midstream urine was gathered into a 20 mL calibration sterilized screw-capped generic container, which has been given to them at the start [2]. Within hours of collection, the sample was properly labeled, transferred to the laboratories, and analyzed. Before collecting the urine specimen, all participants were given detailed instructions on how to take the specimen aseptically to prevent contamination. Furthermore, all patients gave verbal explicit consent to participate in sample collection, as well as the research, carried out after receiving ethical clearance from the hospital management.

### 3.2. Urinary Pathogens

#### 3.2.1. Pathogenic Bacteria

E. coli causes 85% of the population urinary tract infections and 50% of hospital-acquired infections. There are several subtypes of E. coli that are regularly identified from UTI victims. The vast majority of community-acquired illnesses are caused by Gram-negative bacteria such as Klebsiella and Proteus, whereas the remaining infections are caused by Gram-positive bacteria such as Staphylococcus saprophyticus and Enterococcus faecalis. Antibiotics are generally ineffective against Gram-negative bacteria due to their great resistance. They are one of the most significant threats to the world's public health [17]. After being colonized with Pseudomonas aeruginosa, Klebsiella, S. epidermidis, Citrobacter, Serratia, Enterobacter, Providencia, or E. faecalis, the majority of hospital-acquired illnesses generally appear. Importantly, the participant's age may affect the selection of infective bacteria found, with Staphylococcus saprophyticus currently responsible for 10% of UTIs among young girls contrasted with less than 1% in old females.

### 3.3. Uncomplicated and Complicated Urinary Tract Infection

There is widespread agreement that distinguishing between severe and simple infections is critical for the effective therapy of individuals with urinary tract infections. Diseases of the parenchyma, such as glomerulonephritis and prostate disease, are examples of complex infections that frequently manifest themselves in the context of obstructive uropathy or even after catheterization. A clog can cause damage to the kidneys, as well as kidney stones and infection [18]. Kidney injury is predisposed by the incidence of blockage, pebbles, or maximum-pressure vesicoureteric reflux, perinephric abscess, life-severe septicemia, or a mixture as shown in Figure 2. Cycles may be resistant to treatment, producing depressive episodes and, in rare cases, serious complications including infection, metastatic abscesses, and acute renal failure [19]. A period of cystourethritis caused by bacterial colonization of a ureteral and bladder mucosae is known as an uncomplicated disease. Although sequelae are few and limited due to significant morbidity with reinfection in a subgroup of women, this kind of infection is termed simple. Young women having pyelonephritis (diagnosis of acute pyelonephritis) that react well to treatment may have a reduced risk of complications.

#### 3.3.1. Uncomplicated UTI

According to the underlying host variables and underlying uropathogens, UTIs can be classed as difficult or uncomplicated, as shown in Table 1. Over the previous two to three decades, the aetiology of simple UTIs has remained consistent, with an E. coli responsible for the great majority of infections. Earlier, female patients with simple UTIs were often susceptible to trimethoprim-sulfamethoxazole conjunction, and the standard treatment strategy was an experimental short-course antibacterial treatment [20]. Furthermore, a handful of research studies has shown an increase in antibiotic resistance within uropathogens that cause uncomplicated conjunctivitis, raising doubts about standard antibiotic regimens [21]. Throughout a 5-year investigation, researchers looked at antibiotic resistance in 4000 female patients having UTI isolates. According to the findings of this research, the rate of antimicrobial resistance increased from nine percent to eighteen percent when treatment with trimethoprim-sulfamethoxazole was administered to patients. Additionally, resistance to ampicillin climbed from 26 percent to 34 percent, while susceptibility to cephalothin, the first cephalosporin, improved from 20 percent to 28 percent. The resistance to nitrofurantoin and ciprofloxacin, for example, remained at 1% after 5 years. Previous treatment of diabetes mellitus, trimethoprim-sulfamethoxazole, recent hospitalizations, and recent treatment of every other antibiotic have all been linked to the development of resistant bacteria.

Antibiotic regimens typically used to treat simple urinary tract infections may need to be changed as a result of rising resistance patterns [22]. In premenopausal females having uncomplicated pyelonephritis, 7-day treatment of ciprofloxacin was found to have a higher cure rate than a 14-day treatment of trimethoprim-sulfamethoxazole. In this experiment, the proportion of E. coli strains that are resistant to trimethoprim-sulfamethoxazole is significantly higher (18%) than the proportion that is resistant to ciprofloxacin (0%). The antibiotic amoxicillin was found to have the highest risk of E. coli resistance, followed by the antibiotics cefuroxime and ceftriaxone in that order. The research found that females given with trimethoprim-sulfamethoxazole had worse treatment efficacy for uncomplicated UTIs, the overall rate of failure increasing from 3% to 14% in sensitivity E. coli strains as well as from 28% to 40% in resistant organisms. Antimicrobial medication with a fluoroquinolone or, nitrofurantoin, fosfomycin is presently suggested for uncomplicated UTIs depending on this research [1]. Importantly, clinicians should be informed of the antibacterial range of these medicines before administering them, as nitrofurantoin is ineffective for treatment of simple pyelonephritis but extremely successful for acute cystitis. Recurrent uncomplicated UTIs occurred in 25% to 35% of individuals 3 to 6 months following their original UTI. In up to 60% of individuals having recurrent UTI, another stress is produced by a similar straining to an initial.

#### 3.3.2. Complicated UTI

Complicated UTIs are predisposed by underlying host characteristics such as spinal cord damage, catheterization, age, and diabetes mellitus as in Figure 3. Less infectious uropathogens (which hardly cause illness in a healthy urinary system) can produce severe harm to aberrant urinary tract in complex UTIs [23]. In the elderly, studies have found links among Enterococci, Group B streptococcal bacteremia, and Candida, as well as problematic UTIs.

Staphylococcus aureus has been the most often isolated microbe in pediatric patients using indwelling urinary catheters, and adolescents having comorbidities seem to be more prone to have complex UTIs [24]. After instruments of the pediatric urinary bladder, Candida and coagulase-negative staphylococci are linked to complex UTIs. In adolescents with simple UTIs, Enterobacteriaceae is perhaps the greatest frequently identified uropathogen. Uropathogens such as E. coli, Enterococcus, Klebsiella, and Group B Streptococci are some of the top ten aggravating diseases in individuals with diabetes mellitus. In addition, Klebsiella and Group B Streptococcus were 2-3 times less shared in diabetic patients than in those who do not have the disease.

E. coli remained the maximum common uropathogen in people with diabetes having UTIs, as evidenced by prospective research that found E. coli in 56.1% of diabetic patients with UTIs. Patients with diabetes had a greater percentage of bladder catheterization, which could explain the developed occurrence in the patient group [25]. Uropathogens such as E. coli, Pseudomonas, and Proteus mirabilis are common culprits in the development of severe UTIs in patients who have spinal cord injuries and have catheters that remain in place. The E. coli bacteria are a type of bacteria that are typically found in a person's intestines. The latter is linked to difficult UTIs because it has specific virulence characteristics that increase the extent of the problem. Over 9 years, one study found significant growth in nosocomial UTIs, from 2.64 per 1000 patient days to 4.36 per 1000 patient days (*p* < 0.003). Notably, catheter-related UTIs accounted for 88% of nosocomial UTIs in this research. In both complex and mild urinary tract infections (UTIs), basic uropathogens are often isolated as demonstrated in Table 1.  Table 2 shows the bacteria identified from catheterized and noncatheterized patients' urine specimens.

### 3.4. E. coli Pathogenic and Nonpathogenic Types

Type 1 pili were also known as mannose sensitivity pili, seen in both pathogenic and nonpathogenic E. coli types. They are called mannose sensitive because mannose inhibits the hemagglutination of erythrocytes. The helical rod having repeated FimA subunits is attached to the distant structure of tip that contains the FimH adhesin in type 1 pili. FimH adhesins attach to mannosylated sensors on the patient's uroepithelium as carried out on the basis. Following the start of the bond formation, an inflammatory response develops. Several investigations have shown that connections among the FimH adhesin and the epithelial cells upon that bladder's surfaces were required for uropathogenic E. coli strains to colonize and attack the bladder epithelium [26]. Whenever type 1 pili connect to uroplakin 1a (UP1a) and uroplakin 1b (UP1b), a unique “adhesin-epithelial cell” binding mechanism happens (UP1b) in Figure 4. Uroplakins are membrane proteins present on umbrella cells that border the urine bladder's luminal surface. First, adhesin binding processes were studied in the mouse cystitis model, in which a large number of bacteria connected to the urothelial surfaces of a mouse urinary system quickly after infection. FimH-containing pili connected to a body cavity in uroplakin hexametric bands, according to transmission electron microscopy of such urothelial levels; the binding mechanism is essential for the earliest path important to productive UTI.

Activation process FimH adhesins travel to bottomless urothelial levels and enter the membrane following attaching to the epithelial layer. The invading procedure goes once the multiple definitions are intracellular, as bacteria grow within the cytosol to create a network. Eight hours later injection, the bacteria's phenotypic appearance transforms to an enveloping “biofilm”-like structure that defends the uropathogen from the host's immune answer and shelters it from its surroundings in Figure 5. If the rate at which bacteria reproduce can be slowed down, then the creation of a “biofilm matrix” will have a better chance of being successful. The formation of biofilms can be attributed to a variety of factors, all of which contribute to the expansion and maintenance of the microorganisms [27]. This matrix can keep neutrophils from reaching the host's membrane. The theory of a “biofilm” is based on the premise that bacteria work together to stay alive and grow after connecting to a prepared surface. Biofilms have previously been shown to have a significant role in a variety of pathological conditions. Infectious urinary tract Pseudomonas, calculi, infestations in the patients with a cystic fibrosis, and infectious endocarditis can all produce bacterial biofilms [28]. Biofilms create irreversible relationships with their hosts during the illness process by generating external polysaccharides with specialized tasks.

### 3.5. Processing of Samples and Organism Identification

The specimens were analyzed using a methodology that had previously been disclosed. Only participants with pathological changes of UTI and positive urine culture (10^5^ CFU/mL) were involved in this study. On arriving at the hospital, each urine test was inoculated aseptically (in triplicate) into MacConkey agar plates, mannitol salt agar sheets, and cetrimide agar plates [29]. For 18–24 hours, the samples were incubated aerobically at 37°C. The unique isolated strains found on the selective plates contain aseptic conditions subcultured into solution organized in culture medium plates, and the resultant cultures/isolates are microscopically and biochemically tested for accurate diagnosis. The cultural and biochemical belongings of the bacterial separates are utilized to recognize them, as reported in Cheesbrough's famous book. The detected bacterial cultures were kept in the nutrient agar slants for 24 hours, raised at 37°C, and subcultured regularly.

### 3.6. Susceptibility of Antibiotic

The disc distribution method assay is utilized to assess the antimicrobial sensitivity characteristics of isolated bacteria. Nitrofurantoin (NIT) 30 g, ceftazidime (CAZ) 30 g, gentamicin (GEN) 10 g, cefixime (CXM) 5 g, augmentin (AUG) 30 g, ofloxacin (OFL) 5 g, ciprofloxacin (CPR) 5 g, and cefuroxime (CRX) 30 g were all included in the antimicrobial agent (ABTEK, India Seeding Melting Mueller-Hinton agar (MHA)) at 45°C and aseptic conditions pouring into sterilized plates (in triplicate) done using a standardized overnight culture from each isolate [30]. The antibiotic discs were aseptically observed on the top of a growth medium after they had solidified. After that, the MHA samples were maintained at 37°C for 24 hours. The regions of inhibition are evaluated and then analyzed using the Clinical and Laboratory Standards Institute's (CLSI) standards after a 24-hour incubation period.

### 3.7. Multiple Antibiotic Resistance Index (MARI)

By separating the total quantity of antibiotics to a microbe unaffected by the overall range of antibiotics to the organism that has been exposed, the MARI assessment was made [31].

## 4. Result and Discussion

One of the most dominant bacterial infections in the human urinary system is UTI. They are usually treated based on experience, and the criterion for choosing antimicrobial drugs should be created on a most likely disease and its anticipated resistance trend in the area. As a result, periodic observation of the causal organism of UTI, as well as their resistance/susceptibility patterns in a given area, is required. The details of culture characterization are shown in Table 3. 215 bacterial cultures were recovered from the 100 positive urine cultures. S. aureus is discovered to be the most prevalent urinary pathogen followed by E. coli and then a coagulase-negative Staphylococcus species, S. saprophyticus, and S. aureus which was the most frequently identified uropathogen among individuals with clinical symptoms of UTI in earlier research in south-southern Nigeria.

Figure 6 shows the frequency rates of various bacteria identified. Receptive anal activity and HIV infection were blamed for the high incidence of S. aureus. Previously, several researches had connected the rising incidence of Staphylococcus UTIs to greater usage of instruments including bladder catheterization. Nevertheless, the large number of Staphylococcus detected differed from several earlier research in which E. coli was reported to be the most common in UTI. This variance supports the idea in which the distribution of UTI-causing organisms, as well as their antibiotic susceptibility patterns, differs from area to area and through time. Streptococci are not regularly separated but remain important clinical uropathogens. S. saprophyticus has indeed been described as two maximum common cultured uropathogen, although Streptococci are not commonly separated but continue clinically relevant uropathogens. This adds to the study's finding of a minimal concentration of Streptococcus species.

Burckhardt and Zimmermann stated in 2011 that there are few published examples of UTIs caused by Streptococci, although they continued to believe that Streptococci are possible UTI-causing bacteria, particularly among those with urinary tract abnormalities. Urosepsis, asymptomatic bacteriuria (ABU), urethritis, cystitis, and pyelonephritis are all symptoms of Group B Streptococcus UTI. Furthermore, there is presence of Bacillus and Neisseria gonorrhoeae in investigation due to colonization. STD was discovered in 18% of the sexually active women who presented with UTI concerns. They concluded that people with UTI symptoms can have a wide range of STDs.

### 4.1. UTI Prevalence

Patients provided two hundred and fifty-eight (258) fresh-collection midstream urine samples. In 88/258 cases, substantial bacteriuria was found (32.2%). The frequency of bacterial UTI is greatest in a group of age 20–29 years, by 28/88 (32.6%), and lowest in the adolescent age range 10–19 years, with 1/86 (1.2%) as in Table 4.

Females had the highest rate of urinary tract infection, with 66/176 (37.5%) as opposed to 20/91 (22.0%) in men.  Figure 7 shows the blue bar as male, orange bar as female, and gray bar as total. Escherichia coli is the most common bacterial uropathogen including 36/86 (41.9%), tracked by Klebsiella oxytocin 6/86 (7.0%), Staphylococcus aureus 27/86 (31.4%), Klebsiella pneumoniae 10/86 (11.6%), Proteus mirabilis 3/86 (3.5%), Proteus vulgaris 1/86 (1.2%), and Enterococcus faecalis 3/86 (3.5%).

Based on the overall responsiveness of the samples to every antibiotic examined in Table 5, Streptococcus sp. appears to be the most susceptible isolate in this investigation, with excellent susceptibility to every antibiotic studied. All of the microorganisms too were found to be more disposed to nitrofurantoin, ciprofloxacin, and ofloxacin to variable degrees. This is consistent with prior research findings. Nitrofurantoin had the best action against most of the isolated, according to all of them. In the past, ciprofloxacin has shown to be very efficient against uropathogens. Ciprofloxacin has demonstrated exceptional efficacy against uropathogens in the past. Cefuroxime, amoxicillin-clavulanic acid, cefixime, and ceftazidime, along with the majority of the other drugs used exhibited varied degrees of resistance in the primary isolates. This observation is consistent with Uwaezuoke and Ogbulie's findings. Because nitrofurantoin was found to be responsive to a higher proportion of UTI isolated strains in this research, this would be an appropriate candidate for UTI potential therapies whereas awaiting the results of culture and sensitivity testing. The patient's condition, however, may need the use of ciprofloxacin or ofloxacin. Surprisingly, most of the isolated were amoxicillin-clavulanic acid-resistant.

This maximum incidence of amoxicillin-clavulanic acid tolerance is related to the irrational usage of medicine in this area. Antibiotic self-medication, which is routinely used to treat a variety of ailments, has indeed been identified as one key mechanism of generating bacterial resistance. Clavulanic acids within the amoxicillin-clavulanic acid combination are supposed to protect the lactam chemical ring nuclei in the amoxicillin, and the protection must be projected to increase amoxicillin's effectiveness. As a result, an amoxicillin-clavulanic acid combination should have significantly higher susceptibility charges than the isolates. The accessibility and solubility parameters that influence antibiotic transfer through microbial cells are linked to the reported resistance. As a result, because the amoxicillin-clavulanic acid combination is such a big molecule, it may have a difficult time permeabilizing and transporting transversely the bacteriological wall. As a result, increased resistance could be attributed to a comparatively small number of antimicrobial agents accessible. The results on lactams, particularly cephalosporins, are consistent with Saxena's observations.

The MARI's outcome is shown in Figure 8. Always one isolated, Streptococcus spp., had a MARI of less than 0.20 from the MARI collected in this study (0.125). Others rated MARI as being better. MARI is a representation that enables how bacteria resistance spreads in a community. If a MARI is larger than 0.20, bacteria strains were from an atmosphere where many antibiotics were administered or abused. This means that a significant number of the isolated bacteria have been treated with many drugs and have evolved resistance to them. In the research of Ehinmidu (2003), a similar frequency was observed, although not to the same group of medicines. Uropathogens were resistant to routinely utilized antibacterial, according to both [31]. The study's problem would be that the medical studies of the participants (gender, age, catheter-associated UTI, etc.) were not recorded.

## 5. Conclusion

Finally, the discovery of bacteria in UTIs by increased resistance charges to routinely utilized antibacterial drugs leaves physicians with a limited number of alternatives for empirical therapy of UTIs. The most common bacterial uropathogen producing urine infection is E. coli. Among several uropathogens studied, S. aureus, S. saprophyticus, and E. coli have been the most common. The significant MARI of urine specimens isolated in this area emphasizes the importance of continuing to evaluate the antibiotic resistance characteristics of bacteria associated with UTIs before prescribing antibiotics to the highest performance and desirable therapy. However, propose that nitrofurantoin, ciprofloxacin, and ofloxacin be used first in empiric therapy of UTIs in the area. The use of antimicrobial resistance characteristics in the action of UTI and the availability of suitable antibiotics have a lot of potential in the future. Antimicrobial resistance processes appearing in microorganisms from urine samples suggest that UTIs could become more harmful in the future.

## Figures and Tables

**Figure 1:** Patients with an existing UTI are more likely to develop ascending infection pathways.

**Figure 2:** Uncomplicated and complicated UTI classifications.

**Figure 3:** Factors that make complicated UTIs more frequent.

**Figure 4:** FimH adhesins connect to umbrella membranes through uroplakin 1a (UP1a) and uroplakin 1b (UP1b) membrane receptors in colonization.

**Figure 5:** (a) The uropathogenic microorganisms would reach the cytosol following adhering to an epithelial surface. (b) During the first 24 hours, intracellular microorganisms multiply fast. (c) As a result, the rate of growth slows and a protected biofilm matrix emerges. (d) The uropathogen can elude the immunological response of the host by changing its morphology. Aggregated uropathogens become motile and separate from the biofilm, allowing them to disseminate.

**Figure 6:** Frequency rates of various bacteria identified.

**Figure 7:** Identified bacterial uropathogens are common.

**Figure 8:** MARI of bacterial isolates.

**Table 1:** Comparison of complicated and uncomplicated UTI.

Sl. no.	Pathogens in complicated UTI	Pathogens in uncomplicated UTIs
1	E. coli	E. coli
2		Group B Streptococci
3	Staphylococcus saprophyticus	Klebsiella
4		Enterococcus faecalis
5	Klebsiella	Enterobacter cloacae
6		Proteus mirabilis
7	Enterococcus faecalis	Serratia marcescens
8		Pseudomonas aeruginosa

**Table 2:** Bacteria identified from urine specimens.

Microorganism	Catheterized	Noncatheterized	Overall
Klebsiella	20	170	190
Enterococcus faecalis	1	35	97
E. coli	32	688	718
Citrobacter freundii	—	10	10
Staphylococcus saprophyticus	—	27	27
Staphylococcus aureus	1	98	42
Pseudomonas aeruginosa	2	38	36
Proteus mirabilis	10	81	88
Overall	66	1147	1208

**Table 3:** Frequency of bacteria identified from patients' urine specimens.

Bacteria identified	Number of identified bacteria	Frequency rates
E. coli	54	25.7
Staphylococcus saprophyticus	44	21
Staphylococcus aureus	61	29
Pseudomonas aeruginosa	19	8.5
Proteus	10	4.1
Klebsiella	9	3.8
Enterococcus faecalis	11	3.5
Staphylococcus	7	1.7
Bacillus	4	1.4
Neisseria gonorrhoeae	4	1.4
Overall	223	100

**Table 4:** Specific age of bacterial prevalence uropathogens.

Range of age	UTI of positive	UTI of negative	Overall
<1	8	14	22
1-10	6	29	35
11-20	10	20	30
21-30	29	38	67
31-40	12	23	36
41-50	14	21	35
51-60	9	25	34
Overall	88	170	258

**Table 5:** Variation of antimicrobial sensitivity of isolated bacteria from urine samples.

Identifies	E. coli	Staphylococcus saprophyticus	Proteus	Pseudomonas aeruginosa	Staphylococcus aureus	Klebsiella	Enterococcus Faecalis	Staphylococcus	Bacillus
*Gentamicin*									
Susceptible	55.3	29.7	55.7	62	29.7	67.8	84.3	67.8	67.8
Resistant	35.4	67.8	17.8	42	72.5	0	17.6	0	34.3
Moderate sensitive	10.4	4.8	28.9	0	0	34.3	34.3	0	0

*Cefuroxime*									
Susceptible	13.9	4.9	0	0	0	0	0	0	0
Resistant	65.7	82	66.8	71	58	100	16.8	66.8	33.4
Moderate sensitive	21.7	14.5	33.4	32	44	0	84.5	33.4	66.8

*Cefixime*									
Susceptible	35.6	19.1	66.8	62	0	66.8	84.3	67.6	0
Resistant	39	47.5	22.3	42	45	0	16.8	33.4	33.4
Moderate sensitive	28.4	33.4	11.2	0	58	33.4	0	0	66.8

*Ofloxacin*									
Susceptible	52.8	82	73.2	42	71.5	33.4	84.3	100	66.8
Resistant	41.5	14.4	28.9	52	29.7	67.8	17.6	0	33.4
Moderate sensitive	6.8	4.8	0	12	0	0	0	0	0

*Antibiotic amoxicillin-clavulanic acid*									
Susceptible	10.5	9.6	0	0	14.5	0	0	0	0
Resistant	83.5	72.5	95.6	92	86.8	100	100	67.8	67.8
Moderate sensitive	19	6.8	5.1	10	0	0	0	34.3	34.3

*Nitrofurantoin*									
Susceptible	66.8	71	58	100	16.8	66.8	67.8	17.8	42
Resistant	28.9	52	29.7	67.8	17.6	0	0	58	33.4
Moderate sensitive	32	44	0	84.5	33.4	52	29.7	67.8	17.6

*Ciprofloxacin*									
Susceptible	57.9	67.8	73.2	62	86.8	100	100	67.8	0
Resistant	52	29.7	67.8	17.6	58	33.4	0	0	0
Moderate sensitive	3.5	14.5	0	0	0	0	0	0	34.3

*Ceftazidime*									
Susceptible	8	4.9	0	0	14.5	0	34.3	0	0
Resistant	78.9	77.3	0	0	14.5	0	34.3	0	0
Moderate sensitive	17.3	19	39.8	10	14.5	34.5	16.8	33.4	68.7

## Data Availability

The data used to support the findings of this study are included within the article. Further data or information is available from the corresponding author upon request.
